# RAB22A overexpression promotes the tumor growth of melanoma

This article has been retracted.

**DOI:** 10.18632/oncotarget.12329

**Published:** 2016-09-28

**Authors:** Feng Su, Yifei Chen, Shilin Zhu, Fangfang Li, Shuang Zhao, Lisa Wu, Xiang Chen, Juan Su

**Affiliations:** ^1^ Department of Emergency, Xiangya Hospital, Central South University, Changsha, China; ^2^ Department of Pharmacy, Xiangya Hospital, Central South University, Changsha, Hunan, China; ^3^ Department of Neurology, The Second Affiliated Hospital of Hunan University of TCM, Changsha, Hunan, China; ^4^ Department of Dermatology, Xiangya Hospital, Central South University, Changsha, Hunan, China; ^5^ Hunan Key Laboratory of Skin Cancer and Psoriasis, Xiangya Hospital, Central South University, Changsha, Hunan, China; ^6^ Institute of Medical Science Research, Xiangya Hospital, Central South University, Hunan, China

**Keywords:** melanoma, RAB22A, prognosis, malignant phenotype, microRNA

## Abstract

Malignant melanoma is the most aggressive type of skin cancer. RAB22A, a member of RAS oncogene family, has been found to be significantly upregulated in multiple human cancers. In the present study, we found that RAB22A mRNA expression was significantly upregulated in melanoma tissues (including 60 primary melanomas and 84 metastatic melanomas) compared to benign nevi (*n* = 20), which were significantly higher in metastatic melanoma tissues than primary tissues. Immunohistochemistry data further showed that the positive immunoreactivity of RAB22A was detected in 66% (95/144) melanoma tissues, but not in benign nevi. Moreover, high expression of RAB22A was significantly associated with advanced clinical stage in melanoma. Furthermore, patients with high RAB22A expression had shorter overall survival compared those with low expression of RAB22A. In-vitro study showed that RAB22A was also upregulated in melanoma cell lines WM35, A375, WM451, and SK-MEL-1, when compared with the normal melanocyte HM cells. Knockdown of RAB22A significantly reduced the proliferation, migration and invasion of melanoma A375 cells, while overexpression of RAB22A significantly promoted these malignant phenotypes. In addition, RAB22A was found to be a target of miR-203, a tumor suppressive miRNA in melanoma. Besides, miR-203 was downregulated in melanoma tissues and cell lines, when compared with benign nevi and HM cells, respectively. Taken these findings together, our study could validate an oncogenic role of RAB22A in melanoma, suggesting that RAB22A may be a potential therapeutic target for melanoma.

## INTRODUCTION

Malignant melanoma is one of the most aggressive forms of skin cancer in worldwide, with a very poor 5-year survival rate [1]. Moreover, the incidence of melanoma has been increasing in recent decades [2, 3]. Although significant progresses have been made in the early diagnosis and treatment of this disease, the prognosis of melanoma remains poor, mainly due to its recurrence and metastasis as well as lack of efficient biomarkers [3]. Therefore, it is urgently needed to develop novel specific biomarkers for its early diagnosis and treatment. Recently, many oncogenes and tumor suppressor genes have been proved to be deregulated in melanoma, which contribute to its malignant progression [4–8].

RAB22A, a small GTPase that is expressed ubiquitously in mammalian tissues, plays a key role in endosomal membrane trafficking [9]. Overexpression of RAB22A causes a prominent morphological enlargement of the early and late endosomes, but hampers the transport between endosomes and the Golgi apparatus [10, 11]. Recently, RAB22A was found to be frequently upregulated in several human cancers and act as an oncogene [12, 13]. For instance, He et al. reported that RAB22A was significantly upregulated in hepatocellular carcinoma [12]. Yang et al. found that the expression of RAB22A was markedly increased in human osteosarcoma tissues and cell lines [13]. Moreover, RAB22A showed positive expression at the regions of chromosomal breakpoints in malignant melanoma [14]. Knockdown of RAB22A increases the epithelial properties and impairs the mesenchymal properties of the melanoma cells [15], suggesting that RAB22A plays a promoting role in the epithelial mesenchymal transition (EMT), which is essential for tumor metastasis [16].

Recently, the RAB22A expression in human cancers was found to be regulated by epigenetical mechanism, and several microRNAs (miRs) were reported to function as tumor suppressors through directly targeting RAB22A [15, 17, 18]. Xiong et al. showed that miR-204 inhibited the proliferation and invasion of renal cell carcinoma cells by inhibiting the expression of RAB22A [17]. Moreover, Yu et al. reported that MiR-211 inhibited the EMT of melanoma cells by targeting RAB22A [15]. However, whether other miRs directly targeting RAB22A in melanoma exist has not been fully understood. Thus, our study aimed to investigate the clinical significance of RAB22A expression in melanoma, as well as the exact role of RAB22A in the malignant phenotypes of melanoma cells. In addition, we also studied the epigenetical mechanism of RAB22A expression in melanoma cells.

## RESULTS

### RAB22A was overexpressed in melanoma tissue

In the present study, we firstly examined the mRNA expression of RAB22A expression using a RT-qPCR assay. As shown in Figure 1A, the mRNA levels of RAB22A were significantly higher in melanoma compared to those in benign nevi. Moreover, its expression levels were significantly increased in metastatic melanoma tissues compared to those in primary melanoma tissues (Figure 1B).

**Figure 1:** (**A**) Real-time PCR was used to examine the mRNA levels of RAB22A in melanoma compared to benign nevi. **P < 0.01 vs. Nevi. (**B**) Real-time PCR was used to examine the mRNA levels of RAB22A in metastatic melanoma tissues compared to primary melanoma tissues (Figure 1B). **P < 0.01 vs. Primary melanoma. All the experiments were repeated for 3 times.

### RAB22A expression was associated with certain clinicopathologic characteristics in melanoma

As shown in Figure 2, RAB22A protein was expressed mainly in the cytoplasm (brown). Immunohistochemistry data further showed that the positive immunoreactivity of RAB22A was detected in 66% (95/144) melanoma tissues, but no positive immunoreactivity of RAB22A was detected in benign nevi. We further investigated the association between the RAB22A protein expression and clinicopathological characteristics in melanoma cases. According to the protein expression of RAB22A, patients were divided into high expression group (+++ and ++) and low expression group (+ and −). As shown in Table 1, high expression of RAB22A was significantly associated with advanced clinical stage in melanoma (*P* < 0.05), but not with age, sex, family history, ulcer, or occurrence site (all *P* > 0.05). These findings suggest that upregulation of RAB22A may contribute to the malignant progression of melanoma.

**Figure 2:** Representative images of RAB22A immunostaining (**A**) RAB22A expression was not detected. (**B**) RAB22A expression was mainly located in the cytoplasm. (×200 magnification) All the experiments were repeated for 3 times.

**Table 1:** Association between RAB22A expression and clinicopathological characteristics

Variables	Number	Low RAB22A (*n* = 68)	High RAB22A (*n* = 76)	*P* value
**Age**				0.503
< 50	65	33	32	
≥ 50	79	35	44	
**Sex**				0.613
Male	83	41	42	
Female	61	27	34	
**Family history**				0.479
Yes	21	8	13	
No	123	60	63	
**TMN stage**				0.002
I–II	77	46	31	
III	67	22	45	
**Ulcer**				0.872
Yes	61	35	36	
No	83	43	40	
**Occurrence site**				0.313
Trunk + head	82	42	40	
Extremities	62	26	36	

### High expression of RAB22A could predict poor prognosis in patients with melanoma

We then examined the association with RAB22A expression and overall survival time of patients with melanoma. As indicated in Figure 3, patients with high RAB22A expression (+++ and ++) showed shorter survival time, when compared with those with low RAB22A expression (+ and −). These data indicate that high expression of RAB22A was associated with poor prognosis of patients with melanoma.

**Figure 3:** The overall survival curves for melanoma patients with high expression (+++ and ++) and low expression (+ and −) of RAB22A All the experiments were repeated for 3 times.

### Knockdown of RAB22A inhibited the malignant phenotypes of melanoma cells

Western blot data further showed that RAB22A was also upregulated in melanoma cell lines including WM35, A375, WM451, and SK-MEL-1, when compared with the normal melanocyte (HM) cells (Figure 4A). The regulatory role of RAB22A in the malignant phenotypes of A375 was further studied. As RAB22A was significantly upregulated in melanoma, RAB22A-specific siRNA was used to transfect A375 cells to decrease its expression. Transfection with non-specific siRNA was used as the control group. As shown in Figure 4B, the protein levels of RAB22A were significantly lower in RAB22A siRNA group, compared to the control group. The cell proliferation, migration and invasion were further examined. As shown in Figure 4C–4E, knockdown of RAB22A caused a significant decrease in the proliferation, migration and invasion of A375 cells, when compared to the control group, respectively.

**Figure 4:** (**A**) Western blot was conducted to determine the protein levels of RAB22A in melanoma cell lines including WM35, A375, WM451, and SK-MEL-1, when compared with the normal melanocyte (HM) cells. (**B**) Western blot was conducted to determine the protein levels of RAB22A in A375 cells transfected with RAB22A siRNA, or non-specific siRNA as control group. (**C**) MTT assay, (**D**) wound healing assay and (**E**) transwell assay were used to examine the cell proliferation, migration and invasion, respectively. **P < 0.01 vs. Control. All the experiments were repeated for 3 times.

To further confirm our findings, pcDNA3.1-RAB22A ORF plasmid was used to transfect A375 cells to increase its expression. Transfection with blank vector was used as the control group. After transfected with pcDNA3.1-RAB22A ORF plasmid, the protein levels were significantly increased (Figure 5A). Moreover, overexpression of RAB22A significantly upregulated the proliferation, migration and invasion of A375 cells (Figure 5B–5D), when compared with the control group, respectively. These findings indicate that RAB22A plays an oncogenic role in the malignant phenotypes of melanoma cells.

**Figure 5:** (**A**) Western blot was conducted to determine the protein levels of RAB22A in A375 cells transfected with pcDNA3.1-RAB22A ORF plasmid, or blank vector as control group. (**B**) MTT assay, (**C**) wound healing assay and (**D**) transwell assay were used to examine the cell proliferation, migration and invasion, respectively. **P < 0.01 vs. Control. All the experiments were repeated for 3 times.

### RAB22A is a target gene of miR-203, a tumor suppressive miR in melanoma

In addition, we studied the regulatory mechanism of RAB22A in melanoma cells. MiR-203 was previously reported to be significantly downregulated in melanoma, and function as a tumor suppressor. We found that overexpression of miR-203 significantly decreased the protein expression of RAB22A, while knockdown of miR-203 by specific siRNA remarkably enhanced the RAB22A protein expression in melanoma cells (Figure 6). To further clarify their relationship in melanoma, we generated the WT and MT RAB22A 3′UTR reporter plasmids (Figure 7A), and performed luciferase reporter assay. As shown in Figure 7B, the luciferase activity was significantly decreased in A375 cells transfected with miR-203 mimic and WT RAB22A 3′UTR reporter plasmid, which was abolished by MT RAB22A 3′UTR reporter plasmid. Accordingly, RAB22A is a directly target gene of miR-203 in A375 cells. We further investigated the association between the miR-203 and RAB22A expression in melanoma tissues. As shown in Figure 7C, real-time PCR data indicated that miR-203 was significantly downregulated in melanoma tissues compared with benign nevi. Besides, its expression levels were also reduced in melanoma cell lines compared with HM cells (Figure 7D). These findings suggest that the downregulation of miR-203 may contribute to the upregulation of RAB22A in melanoma cells.

**Figure 6:** (**A**) Real-time PCR was used to examine the miR-203 levels in A375 cells transfected with miR-203 mimic or scramble miR mimic (miR-NC), and then (**B**) western blot was used to examine the protein expression of RAB22A. **P < 0.01 vs. miR-NC. (**C**) Real-time PCR was used to examine the miR-203 levels in A375 cells transfected with miR-203 inhibitor or negative control (NC) inhibitor, and then (**D**) western blot was used to examine the protein expression of RAB22A. **P < 0.01 vs. NC inhibitor. All the experiments were repeated for 3 times.

**Figure 7:** (**A**) The wild type (WT) and mutant type (MT) of RAB22A 3′UTR reporter plasmids were generated. (**B**) The luciferase activity was significantly decreased in A375 cells transfected with miR-203 mimic and WT-RAB22A-3′UTR reporter plasmid, which was abolished by MT-RAB22A-3′UTR reporter plasmid. (**C**) Real-time PCR was used to examine the miR-203 levels in melanoma tissues and benign nevi tissues. **P < 0.01 vs. Nevi. (**D**) Real-time PCR was used to examine the miR-203 levels in melanoma cell lines including WM35, A375, WM451, and SK-MEL-1, when compared with the normal melanocyte (HM) cells. **P < 0.01 vs. HM. All the experiments were repeated for 3 times.

## DISCUSSION

The exact role of RAB22A in melanoma remains largely unclear. In the present study, we found that RAB22A was significantly upregulated in melanoma tissues compared to benign nevi, and also in metastatic melanoma tissues compared to primary tissues. Moreover, high expression of RAB22A was associated with the malignant progression and poor prognosis in melanoma. *In vitro* study showed that RAB22A plays a promoting role in melanoma cell proliferation, migration and invasion. Besides, we suggest that the upregulation of RAB22A in melanoma may be due to the decreased expression of miR-203, which could directly target RAB22A.

Recently, the oncogenic role of RAB22A has gradually been revealed [19, 20]. The expression of RAB22A was found to be significantly upregulated in several cancer types such as hepatocellular carcinoma, osteosarcoma, and colon cancer [12, 13, 21]. Moreover, Wang et al. found that RAB22A was involved in the formation of microvesicles, which could stimulate breast cancer invasion and metastasis [19]. Knockdown of RAB22A reduces the proliferation of gastric cancer cells, suggesting that RAB22A may become a promising molecular target for cancer treatment [20]. Until now, however, the expression as well as the clinical significance of RAB22A in melanoma still remains unknown. Here we firstly found that the mRNA expression of RAB22A was significantly increased in melanoma tissues than benign nevi tissues. Besides, its mRNA levels were also higher in metastatic melanoma tissues compared to primary tissues, suggesting that RAB22A is involved in melanoma development and metastasis. Indeed, immunohistochemical staining data further showed that high expression of RAB22A was significantly associated with advanced clinical stage in melanoma, but not with age, sex, family history, ulcer, or occurrence site. Then, survival analysis indicated that the melanoma patients with high expression of RAB22A had a worse prognosis when compared with those with negative and low expression of RAB22A. Therefore, RAB22A is significantly associated with the malignant progression and poor prognosis in melanoma.

Based on these findings above, we speculated that RAB22A might play a promoting role in the malignant phenotypes of melanoma cells. To verify this speculation, we performed in-vitro experiments using melanoma cell lines. We found that the RAB22A protein levels were also significantly increased in melanoma WM35, WM451, A375, and SK-MEL-1 cell lines, when compared with the normal melanocyte HM cells, consistent with the *in vivo* data. As A375 cells showed the most significant increase in RAB22A expression, we used this cell line in the following studies. We then applied RAB22A-specific siRNA to knockdown the RAB22A expression in A375 cells, and found that inhibition of RAB22A markedly suppressed the proliferation, migration and invasion of A375 cells. Further investigation showed that overexpression of RAB22A indeed promoted these malignant phenotypes of A375 cells, which confirmed our speculation.

MicroRNAs (miRs) are a kind of short non-coding RNAs and can bind to the 3′-untranslational region (UTR) of their target genes, causing mRNA degradation or translation inhibition [22]. MiRs have been found to participate in various biological processes, including cell proliferation, differentiation, apoptosis, migration, and tumorigenesis [22, 23]. In this study, we found that RAB22A was a direct target gene of miR-203, and its protein expression was negatively regulated by miR-203 in A375 cells. MiR-203 has previously been reported to play a suppressive role in melanoma [7, 8, 24, 25]. It is downregulated in melanoma tissues, which is associated with the poor prognosis of melanoma patients [24], and loss of miR-203 expression at the invasive front of primary cutaneous melanoma is associated with increased thickness and disease progression [8], Moreover, miR-203 also has inhibitory effects on the proliferation, migration, and invasion of melanoma cells via targeting versican and BMI1 [7, 25]. Besides, it also can induce senescence in human melanoma cells by inhibiting the protein expression of E2F3 [26]. In this study, we also found that miR-203 was significantly downregulated in melanoma tissues and cell lines, when compared with benign nevi and HM cells, respectively. These findings suggest that the upregulation of RAB22A in melanoma may partly be due to the decreased expression of miR-203. In fact, the targeting relationship between miR-203 and RAB22A was also reported in osteosarcoma [13]. Therefore, our study expands the importance of miR-203/RAB22A axis in human cancers.

In summary, our study demonstrates that RAB22A, significantly upregulated in melanoma, plays an oncogenic role in the malignant phenotypes of melanoma cells, and its expression in melanoma is regulated by epigenetical mechanism. Therefore, RAB22A may be used as a potential therapeutic target for melanoma.

## MATERIALS AND METHODS

### Tissue collection

This study was approved by the legislation and ethical boards of Xiangya Hospital. A total of 144 melanoma tissues (including 60 primary melanomas and 84 metastatic melanomas) and 20 benign nevi were also collected from April 2010 to September 2011. The melanoma tissue was collected before the patients received any treatments including chemotherapy and target therapy. All informed consents were obtained. The tissues were confirmed by the original histopathological and clinical diagnosis. The clinicopathologic characteristics of melanoma cases were summarized in Table 1. No patients received pre-operative chemotherapy or radiotherapy. Tissues were immediately snap-frozen in liquid nitrogen after surgical removal, and stored at −80°C before use.

### Immunohistochemical staining assay

Four μm sections were deparaffinized and subjected to heat-induced antigen retrieval using citrate buffer for 22 min. Then, the sections were incubated with RAB22A antibody (Abcam, USA), and then with the biotinylated secondary antibody (Abcam, USA) for 1 h at room temperature. The reaction was developed using substrate diaminobenzidine (DAB) and counterstained with hematoxylin, and visualized via optical microscopy. For evaluating the expression of RAB22A, all tissue sections were scored independently by three experienced pathologists. The scoring system was as follows: the percentage of positively staining cells was graded as - (negative), +: > 0 and ≤ 25% of cells positive, ++: > 25 and ≤ 75% of cells positive, +++: > 75% of cells positive.

### Cell culture

Human malignant melanoma cell lines WM35, WM451, A375 and SK-MEL-1, and the human melanocyte (HM) cells were obtained from the Cell Bank of Central South University, Changsha, China. Cells were cultured in DMEM supplemented with 10% fetal bovine serum (FBS) at 37°C in a humidified incubator containing 5% CO_2_.

### Cell transfection

Cells were cultured into 70% confluence. RAB22A siRNA (Santa Cruz, USA), non-specific siRNA (Santa Cruz), pcDNA3.1-RAB22A ORF plasmid, blank pcDNA3.1 vector, miR-203 mimic, scramble miR-203, anti-miR-203 (5′-TAGTGGTCCTAAACATTTCA-3′) or Lipofectamine 2000 (Thermo Fisher, USA) was diluted with serum-free medium, respectively. The diluted Lipofectamine 2000 was then added into the diluted siRNA, plasmid or miR at a final concentration of 50 nM, and incubated for 20 min at room temperature, and then added into the cell medium. Then, cells were incubated at 37°C, 5% CO2 for 6 h. After that, the medium was replaced by the DMEM with 10% FBS, and cultured for 24 h before the following assays for expression.

### RNA extraction and real-time RT-PCR

After 12-h transfection, cells were collected and total RNA from cells and tissue was extracted by Ambion RNA isolation kit (Life Technologies, USA). Total miRNAs were extracted using the Ambion mirVana miRNA isolation kit (Life Technologies, USA), and the miRNAs were reverse transcribed with the QuantiMir RT kit (SBI). Real time RT-PCR was conducted to detect the mRNA level of RAB22A or miR-203 using SYBR^®^ GreenMastermix kit (Bio-Rad Laboratories, Hercules, CA) p, and β-actin and U6 were used to be normalized as internal control. Primers were used as following: RAB22A (forward) 5′-TTGTAGCCATTGCAGGA-3′ and (reverse) 5′- AGGCTGTCTTCGGAGTTTGA-3′.

### Western blot

Cells were collected at 48 h after transfection and solubilized in cold RIPA lysis buffer. Proteins (30 μg) were separated with 12% SDS-PAGE, and transferred onto a polyvinylidene difluoride membrane. The membrane was incubated with TBST containing 5% skimmed milk at 37°C for 2 h. After washed with PBST for 3 times, the membrane was incubated with 1:1000 primary anti-RAB22A antibodies (Abcam, USA) at room temperature for 2 h. After washed by PBST for 3 times, the membrane was incubated with 1:2000 secondary antibodies at 4°C overnight. After washed by PBST for 3 times, ECL kit (Pierce Chemical, Rockford, IL, USA) was used to perform chemiluminent detection. Image-Pro plus software 6.0 was used to analyze the relative protein expression, represented as the density ratio versus GAPDH.

### MTT assay

For detection of cell proliferation, 10000 cells per well were plated in a 96-well plate, which were then incubated at 37°C, 5% CO2 for 0, 24, 48 or 72 h, respectively. Then, 10 μL of MTT in PBS (5 mg/ml) was added to each well, and incubated at 37°C, 5% CO2 for 4 h. Then, the supernatant was removed, and 100 μL of DMSO was added. The absorbance was detected at 570 nm with a Microplate Reader (Model 680, Bio-Rad, USA).

### Wound healing assay

A375 cells were cultured to full confluence. Mitomycin C was used to pretreat cells for 2 h. Wounds of approximately 1 mm width were created with a plastic scriber, and cells were washed. After incubated at 37°C, 5% CO2 for 48 h, cells were washed with PBS and observed under microscope.

### Cell invasion assay

For cell invasion assay, 24-well transwell chambers (Chemicon, CA, USA) that has a layer of matrix gel were used. A375 cell suspension (500000 cells/ml) was prepared in serum free DMEM, and 300 μL of cell suspension was added into the upper chamber. Then, 500 μL of DMEM with 10% FBS was added into the lower chamber. After incubation at 37°C with 5 % CO2 for 24 h, cells through the membrane were stained and counted under the microscope.

### Luciferase reporter assay

WT (Wild Type) and MT (mutant) RAB22A 3′UTR reporter plasmids were constructed and cloned into pGL4.10-basic reporter vector. The reporter vectors were cotransfected into A375 cells by Lipofectamine 2000 as the protocol described, and the luciferase reporter activity was detected after 24-h transfection.

### Statistical analysis

All the experiments were triplicated. Continuous variables were expressed as mean ± SD. Statistical analysis of differences *in vitro* study was performed by student *t* test or one-way analysis of variance. Statistical analysis of differences in overall survival time was performed using log-rank tests. *P* < 0.05 was considered statistically significant.
